# Comparison of Pharmacokinetic Profiles of 14 Major Bioactive Components in Normal and Arthritic Model Rats after Oral Administration of *Angelicae pubescentis* Radix by UPLC-MS/MS

**DOI:** 10.1155/2022/8379921

**Published:** 2022-08-16

**Authors:** Ajiao Hou, Huan Yu, Song Wang, Jiaxu Zhang, Xuejiao Wang, Senwang Zheng, Liu Yang, Haixue Kuang, Hai Jiang

**Affiliations:** Key Laboratory of Basic and Application Research of Beiyao, Heilongjiang University of Chinese Medicine, Ministry of Education, Harbin 150040, China

## Abstract

An ultraperformance liquid chromatography tandem mass spectrometry (UPLC-MS/MS) method was established to simultaneously determine 14 compounds of *Angelicae pubescentis* Radix (APR) in normal and arthritis rat plasma in which chloramphenicol and daidzein were used as the internal standards. After protein precipitation with acetonitrile, separation was carried out on a Thermo Hypersil GOLD C_18_ column using gradient elution with 0.1% formic acid aqueous and acetonitrile consisting as the mobile phase at a flowing rate of 0.3 mL/min. A Thermo TSQ QUANTIS triple quadrupole mass spectrometer was used to detect 14 compounds in positive/negative ion exchange mode and this study was the first to investigate the pharmacokinetic changes of the active compounds in rats under the pathological state of arthritis. The method was verified and the results showed that the intra- and interday precision, accuracy, matrix effect, and extraction recovery were all acceptable, and the analytes were stable under different storage conditions. In addition, the pharmacokinetic behaviors of the 14 compounds were significantly different in model rats compared with normal rats. This indicated that the pharmacokinetic behavior of drugs will vary with the pathological state of the body, which suggested that individualized and reasonable drug administration plans should be formulated for different pathological states in clinical practice. This study provided a scientific basis and data support for better understanding the pharmacodynamic substance basis and clinical application of APR against arthritis.

## 1. Introduction

Arthritis generally refers to the inflammatory diseases caused by inflammation, infection, degeneration, trauma, or other factors that occur in the joints and surrounding tissues of the human body [1]. The clinical manifestations include joint redness, swelling, pain, dysfunction, and joint deformity, which will lead to joint disability and affect the quality of life of patients in severe cases [2]. According to statistics, there are more than 100 million people who suffer from arthritis in China; the prevalence rate is 0.34%–0.36%, and the number is increasing, the life expectancy of severe cases is shortened by about 10–15 years [3]. Modern medicine mostly uses corticosteroids, nonsteroidal anti-inflammatory drugs, immune inhibitors, and disease targeting inhibitors to reduce the degree of joint pain and swelling and delay the development of the disease [4–7]. However, although these drugs have achieved some therapeutic benefits, they can cause serious side effects, weaken the function of the immune system, and increase the risk of infection and are too expensive for patients to bear [8, 9]. Therefore, it is an urgent problem for scientists to find more safe and effective new antiarthritic drugs.

As is known to all, traditional Chinese medicine (TMC) plays an important role in clinical treatment because of its abundant resources, suitable price, stable pharmacological action, low toxicity, and few complications, and some TCMs with antiarthritic effects have been gradually approved for clinical use and have convincing efficacy [10–12]. *Angelicae pubescentis* Radix (APR), a member of the *Apiaceae* family, is the dry root of *Angelica pubescens* Maxim. f. *biserrata* Shan et Yuan. It has the functions of removing wind and dehumidification and relieving paralytic pain [13]. Clinically, it has a good clinical effect on arthritis [14]. In addition, modern pharmacological studies have shown that APR also has anti-inflammatory, antirheumatic, sedative, hypnotic, and neuroprotective effects [15] and contains a variety of chemical components, such as coumarins, phenolic acids, terpenoids, volatile oils, and polysaccharides [13]. Among them, coumarin compounds are one of the main active ingredients of APR to play an antiarthritic role [16–18]. In addition, some studies have shown that phenolic acid compounds also have a certain anti-inflammatory effect [19]. However, the current research study on the antiarthritic effect of APR is limited to the level of pharmacodynamics and pharmacodynamic material basis, and there are few pharmacokinetic studies of its active components, and most of the pharmacokinetic studies of APR have been conducted in normal experimental animals [13, 15, 20, 21]. For example, Qian et al. used HPLC-DAD to determine columbianetin in normal rat plasma [22]. Chang et al. used the LC-MS/MS method to simultaneously determine scopoletin, psoralen, bergapten, xanthotoxin, columbianetin acetate, imperatorin, osthol, isoimperatorin of the AP extract in normal rat plasma [21]. Li et al. used the LC-MS/MS method to simultaneously determine columbianadin and its metabolite columbianetin in rat plasm [23]. However, it is worth noting that there are no pharmacokinetic studies on phenolic acid compounds in AP. The possible reason is that the content of phenolic acid compounds is low in AP, and the lower limit of detection of general detector is not up to the requirement so that phenolic acid compounds cannot be detected. For high-resolution mass spectrometry with lower limit of detection, the researchers may use a single positive ion mode to scan coumarin compounds, which excludes phenolic acids that respond better in negative ion mode. Therefore, we established an UPLC-MS/MS method with positive and negative ion exchange scanning mode for the simultaneous determination of phenolic acids and coumarin compounds [13, 14].

Pharmacokinetics of TCMs is an indispensable link in the modernization of Chinese medicinal materials and an important means of integrating TCMs with the world [24]. Only when the drug reaches a sufficient concentration at the action site in *vivo* can it exert its efficacy, and the plasma drug concentration is not only related to the dosage but is also affected by the process in *vivo*. Moreover, the pharmacokinetic studies of TCMs are mostly carried out based on healthy experimental animals, ignoring the physiological and pathological changes, which may cause significant changes in relevant pharmacokinetic parameters [25, 26]. Studies have shown that the pharmacokinetic characteristics of many drugs in normal and pathological states are different. Under pathological conditions, drug metabolism enzymes, cell membrane permeability, and intestinal flora may change, which further lead to changes in pharmacokinetic parameters [27–31]. The final audience of drugs is disease patients. The body in the pathological state has varying degrees of influence on the absorption, distribution, metabolism, and excretion of drugs, which is closely related to the safety and effectiveness of clinical drug use. Therefore, it is more objective, accurate, and of practical significance for evaluating the pharmacokinetic behavior of the active ingredients of TCMs in model animals than in healthy animals. Furthermore, to our knowledge, no studies have been conducted to compare pharmacokinetic parameters of the active ingredients in normal and arthritic rats after oral administration of APR.

Therefore, a UPLC-MS/MS method was established for simultaneous determination of phenolic acids and coumarin compounds in plasma. This is the first study to investigate the pharmacokinetic change rule of active ingredients of APR in rats with arthritis, so as to provide reference for rational use of drugs in clinical treatment of arthritis.

## 2. Materials and Methods

### 2.1. Chemical Materials

HPLC grade methanol and acetonitrile were obtained from Fisher Scientific (USA). HPLC grade formic acid was purchased from Dikma Co. (USA), and Wahaha purified water was obtained from Hangzhou Wahaha Group (China). Neochlorogenic acid, chlorogenic acid, cryptochlorogenic acid, isochlorogenic acid B (3,4-diCQA), isochlorogenic acid A (3,5-diCQA), isochlorogenic acid C (4,5-diCQA), bergapten, columbianetin acetate, isoimperatorin, osthol, and columbianadin were obtained from Chengdu Must Biotechnology Co., LTD (China), and columbianetin, xanthotoxin, psoralen, and chloramphenicol were obtained from Shanghai Nature Standard Biotechnology Co., LTD (China), and daidzein was obtained from Chengdu Purechem-Standard Biotechnology Co., LTD (China). The purity of the involved standards and reagents were over 98%, with their chemical structures exhibited in Figure 1.

The APR samples was obtained from Hubei Province (30°24N, 115°30E) picked in April 2019, and identified by Professor Lianjie Su from Heilongjiang University of Chinese Medicine, as the dry root of *Angelica pubescens Maxim. f. biserrata* Shan et Yuan and a voucher specimen were deposited at department of Chinese herbal medicine processing of Heilongjiang University of Chinese Medicine, Harbin, China (voucher numbers: APQH201904-7).

### 2.2. Preparation of APR Samples for Rat Administration

One hundred grams of the APR sample was extracted by reflux with 800 mL 50% ethanol/water (v/v) for 3 times (2 hours each time), then combined with the filtrate and concentrated under vacuum with heat, and the concentration of APR extract was 0.37 g/mL. All the sample solutions were stored at 4°C before analysis. The contents of 14 compounds were 61.85 *μ*g/g for neochlorogenic acid, 3006.87 *μ*g/g for chlorogenic acid, 75.08 *μ*g/g for cryptochlorogenic acid, 72.07 *μ*g/g for 3,4-diCQA, 341.27 *μ*g/g for 3,5-diCQA, 112.30 *μ*g/g for 4,5-diCQA, 369.02 *μ*g/g for columbianetin, 3375.11 *μ*g/g for psoralen, 345.41 *μ*g/g for xanthotoxin, 241.69 *μ*g/g for bergapten, 10280.43 *μ*g/g for columbianetin acetate, 25.03 *μ*g/g for isoimperatorin, 7943.10 *μ*g/g for osthol, and 1442.12 *μ*g/g for columbianadin, respectively.

### 2.3. Animal Experiments

Male Sprague-Dawley rats weighing 240–260 g were obtained from the Experimental Animal Center of Heilongjiang University of Chinese Medicine (Harbin, China, Certificate No. SCXK(Hei)2020-0924), and were housed under a room at temperature of 25 ± 2°C and humidity of 50 ± 15%, as well as light/dark circulation, ad libitum access to food and water for more than a week. Moreover, the rats fasted overnight before the experiment. Moreover, the study was authorized by the Ethics Regulations of Heilongjiang University of Chinese Medicine (Harbin, China).

Twelve SD rats were randomly divided into two groups (*n* = 6) and named as the model group and the normal group, respectively. The arthritic model was established by injecting 0.1 mL of complete Freund's adjuvant in rats. As a control, 0.1 mL of saline was injected. After 7 days, the plasma levels of MDA and TNF-*α* in normal and model rats were measured by an enzyme-linked immunosorbent assay kit to determine whether the modeling was successful. The results are shown in Figure 2. The levels of MDA and TNF-*α* in model rats were significantly higher than those in normal rats, indicating that the arthritis model was successfully established. Normal and model rat blood samples were collected from the angular vein at 0.083, 0.167, 0.25, 0.5, 1, 2, 4, 6, 8, 10, 12, 24, 36, and 48 h into 1.5 mL heparinized tubes after administration the APR extract at a dose of 4.1 mL/kg. All samples were immediately centrifuged at 12,000 × g for 15 min at 4°C, and the supernatant was transferred to another EP tube and stored at −80°C until analysis.

### 2.4. Instrumentation and Analytical Conditions

The ultrahigh performance liquid chromatography (Thermo Scientific™, Vanquish™, (Waltham, MA, USA)) was used for the chromatographic analysis. UPLC separation was achieved on a Thermo Hypersil GOLD C_18_ column (100 mm × 2.1 mm, 1.9 *μ*m), which was maintained at 35°C. The mobile phase consisted of 0.1% formic acid aqueous (solvent A) and acetonitrile (solvent B) and the following gradient was run: 7–8% B at 0–4 min, 8–19% B at 4–5 min, 19–19% B at 5–12 min, 19–60% B at 12–15 min, and 60–100% B at 15–18 min, in which the flow rate was maintained at 0.3 mL/min.

The UPLC was interfaced to a Thermo TSQ QUANTIS triple quadrupole mass spectrometer and equipped with an electrospray ionization (ESI) probe working in positive and negative ion exchange scanning mode. The mass spectrum parameters of 14 compounds and their internal standard (IS) compounds were neochlorogenic acid *m/z* 353.0⟶190.9, chlorogenic acid *m/z* 353.0⟶126.9, cryptochlorogenic acid *m/z* 353.0⟶178.9, 3,4-diCQA *m/z* 515.0⟶353.0, 3,5-diCQA *m/z* 515.0⟶191.0, 4,5-diCQA *m/z* 515.0⟶172.9, columbianetin *m/z* 247.0⟶215.0, psoralen *m/z* 187.0⟶143.0, xanthotoxin *m/z* 217.0⟶161.0, bergapten *m/z* 217.0⟶174.0, columbianetin acetate *m/z* 289.0⟶229.0, isoimperatorin *m/z* 271.0⟶239.0, osthol *m/z* 245.0⟶188.9, columbianadin *m/z* 329.0⟶229.0, chloramphenicol *m/z* 321.0⟶257.0, and daidzein *m/z* 254.8⟶198.9. The following parameters were used: sheath gas: 30 Arb; aux gas: 10 Arb; ion transfer tube temp: 325°C; and vaporizer temperature: 350°C.

### 2.5. Standard Solutions, Calibration Standards, and Quality Control (QC) Samples

The standard stock solution of 14 compounds was prepared by dissolving 1 mg of the standard material in 1 ml of methanol, respectively. Then, calibration curve samples were prepared by diluting with different volumes of 50% methanol aqueous to obtain the mixed standard solution. For analysis, aliquots of 100 *μ*L plasma sample and 100 *μ*L mixed standard solution and 20 *μ*L ISs solution were blended with 780 *μ*L acetonitrile, vortexed for 1 min, and the sample solution was immediately centrifuged and separated at 12,000 × g for 15 min at 4°C. At last, the supernatant was removed and placed in another EP tube, where it was dried by nitrogen at 45°C, the residue was dissolved with 100 *μ*L 50% aqueous methanol for UPLC-MS/MS analysis.

Similarly, the three different concentrations of QC samples were obtained at the final concentrations of 10, 252, 504 ng/mL for neochlorogenic acid, 10.6, 1060, 3180 ng/mL for chlorogenic acid, 11.7, 117, 234 ng/mL for cryptochlorogenic acid, 11.2, 56, 112 ng/mL for 3,4-diCQA, 12.5, 312.5, 625 ng/mL for 3,5-diCQA, 20.4, 102, 204 ng/mL for 4,5-diCQA, 39, 2260, 4520 ng/mL for columbianetin, 5.05, 252.5, 505 ng/mL for psoralen, 11.2, 560, 1120 ng/mL for xanthotoxin, 13, 340, 680 ng/mL for bergapten, 54, 2160, 4320 ng/mL for columbianetin acetate, 8.9, 445, 890 ng/mL for isoimperatorin, 5.5, 2200, 5500 ng/mL for osthol, and 12.2, 1220, 2440 ng/mL for columbianadin. In addition, ISs solution with a concentration of 100 ng/mL was used for further analysis, and all the standard solutions, calibration standards, and QC samples were stored at −80°C until further analysis.

### 2.6. Sample Preparation

Acetonitrile was used as a precipitation solvent, and protein precipitation was used to handle with the plasma samples. First, 100 *μ*L aqueous methanol solution and 20 *μ*L ISs solution were added to aliquots of 100 *μ*L of plasma sample following mixing with 780 *μ*L of acetonitrile, and they were centrifuged at 12,000 × g for 15 min at 4°C after being vortexed for 1 min to obtain the supernatant. Then, the supernatant was dried in a nitrogen environment at 45°C, and the remaining residue was recombined with 100 *μ*L 50% methanol aqueous and vortex for 1 min. Finally, 2 *μ*L supernatant was injected into the UPLC-MS/MS system for analysis.

### 2.7. Method Validation

The established UPLC-MS/MS method for the determination of 14 compounds in rat plasma has been validated according to FDA Bioanalytical Method Validation guidelines and the following parameters were evaluated, including selectivity, linearity, sensitivity (LLOQ), precision, accuracy, matrix effect, recoveries, and stability.

#### 2.7.1. Selectivity

Six different individual blank plasma samples not treated with APR, six blank plasma samples with spiked of standards and ISs and six rat plasma samples after oral administration of APR extract 5 min were analyzed by comparison of their corresponding chromatograms to evaluate the selectivity of the method.

#### 2.7.2. Linearity of the Calibration Curve and LLOQ

Calibration curves were established by plotting the ratio of peak area of the individual compound to IS versus different levels of compound with a weighted (1/*χ*^2^) least square linear regression. The lower limit of quantification (LLOQ) was used to represent the sensitivity of the analytical method. Relative error (RE%) and relative standard deviation (RSD%) were used to describe the accuracy and precision, respectively, and both were permitted to be less than ± 20%.

#### 2.7.3. Precision and Accuracy

The intra- and interday precision and accuracy were tested by LLOQ, LQC, MQC, and HQC samples in six replicates on the same day and three successive days. According to FDA guidelines, accuracy and precision for QC samples should not exceed ±15%.

#### 2.7.4. Recovery and Matrix Effect

The extraction recoveries of 14 compounds were evaluated by comparing the peak areas of analyte from blank plasma samples spiked with standards before extraction with post-extraction blank plasma samples spiked with standards at three QC levels. The matrix effect was investigated by comparing peak areas of post-extraction blank plasma samples spiked with standards with the neat solution containing the 14 compounds at the equivalent concentrations.

#### 2.7.5. Stability

The stability of 14 compounds was assessed by LQC, MQC, and HQC in six replicates under different storage conditions: short term stability (room temperature for 4 h), freeze-thaw cycle's stability (three cycles of freeze-thaw), long term stability (storage at −80°C for 30 days), and the posttreatment stability (auto-sampler at 4°C for 24 h).

### 2.8. Pharmacokinetic Study

The pharmacokinetic parameters of 14 compounds including the maximum plasma concentration (*C*_max_), area under concentration-time curve (*AUC*_0–t_ and *AUC*_0-∞_), half-time (*t*_1/2_), time to reach the maximum concentration (*t*_max_), mean retention time (MRT), and clearance rate (CL) were calculated by DAS 2.0 software (Mathematical Pharmacology Professional Committee of China, Shanghai, China) in a noncompartment model.

### 2.9. Statistical Analyses

All data in this study were expressed as mean ± standard deviation (SD). Statistical software GraphPad Prism 5.0 was used for plotting and statistical analysis, and *T* test was used for intergroup comparison. ^*∗*^*P* < 0.05 was considered statistically significant, ^*∗∗*^*P* < 0.01 was considered statistically significant.

## 3. Result and Discussion

### 3.1. Optimization of the Method Conditions

The chromatographic column, mobile phase composition, and elution gradient were optimized in this study in order to achieve the ideal results of the chromatographic behaviors, like good peak symmetry, efficient separation, and short chromatographic retention time. Thermo Hypersil GOLD column (100 mm × 2.1 mm, 1.9 *μ*m) and Waters Acquity UHPLC HSS *T*_3_ column (50 mm × 2.1 mm, 1.8 *μ*m) were used for analysis. The results showed that Thermo Hypersil GOLD column (100 mm × 2.1 mm, 1.9 *μ*m) could detect all compounds in APR with a good peak shape and good separation. Because the coumarin compounds were small polar compounds, and the elution ability of acetonitrile solution was stronger than methanol solution, when methanol solution was used as the mobile phase, the elution time would be prolonged, while acetonitrile solution was used as the mobile phase, greatly shorten the elution time and save solvent. Therefore, acetonitrile was selected as the mobile phase for gradient elution. As neochlorogenic acid, chlorogenic acid, and cryptochlorogenic acid were isomers and difficult to separate, 7% acetonitrile was selected as the initial mobile phase to achieve the best separation effect.

In addition, the mass spectrometry conditions of 14 compounds and ISs compounds were optimized, and the results showed that c, 3,4-diCQA, 3,5-diCQA, 4,5-diCQA, and chloramphenicol (IS_1_) had a better response in negative mode, and bergapten, columbianetin acetate, isoimperatorin, osthol, columbianadin, columbianetin, xanthotoxin, psoralen, and daidzein (IS_2_) had a better response under positive mode.

Sample preparation was one of the most important links in pharmacokinetic research. Compared with expensive solid-phase extraction and complicated liquid-liquid extraction, protein precipitation was a time-saving, economical, and simple method for sample preparation. Therefore, we optimized the precipitation solvents such as methanol, acetonitrile, and ethyl acetate, among which acetonitrile as the precipitation solvent had the best extraction effect on 14 compounds and ISs; so, acetonitrile was finally selected as the precipitation solvents for sample preparation in this study.

### 3.2. Method Validation

#### 3.2.1. Selectivity

The representative chromatograms in three different conditions were as follows: the blank plasma samples, blank plasma samples with spiked of standard and ISs, and the rat plasma after oral APR extract are shown in Figure 3. The result showed that there was no endogenous interference in the retention time of 14 compounds and ISs.

#### 3.2.2. Linearity and LLOQ

The linear regression curve of 14 compounds was verified and it showed excellent linearity within the corresponding concentration range. In this study, the LLOQ for 14 compounds ranged from 0.6 ng/mL to 10.7 ng/mL, with acceptable accuracy and precision, RE <13.84% and RSD value within 14.22%. The linear regression curve, linearity ranges, correlation coefficients, LLOQ are listed in Table 1, and the accuracy and precision of LLOQ of 14 compounds are shown in Table 2.

#### 3.2.3. Precision and Accuracy

The results of the intra- and interday precision and accuracy at three different QC concentration levels are displayed in Table 2. The intra- and interday precision of 14 compounds were in the range of 0.39 to 9.14% and 0.17 to 13.81%, respectively. The accuracy for intra- and interday *r* were in the range of −14.76 to 12.28% and −14.83 to 13.67%, respectively. It illustrated that the method was accurate and precise.

#### 3.2.4. Recovery and Matrix Effect

The extraction recovery and matrix effect were investigated at three different QC concentration levels. The extraction recovery of 14 compounds was in the range of 90.38 ± 7.27% to 103.73 ± 2.78%. The matrix effects of 14 compounds ranged from 88.11 ± 5.31% to 102.29 ± 8.50%, showing that there was basically no interference from endogenous substances. Besides, the extraction recoveries of IS_1_ and IS_2_ were 96.68 ± 2.07% and 99.74 ± 6.36%, respectively. The matrix effect of IS_1_ and IS_2_ were 97.72 ± 3.17% and 99.75 ± 1.89%, respectively. All results are mentioned in Table 3.

#### 3.2.5. Stability

The stability of 14 compounds was measured by QC samples in six replicates under the room temperature for 4 h, three cycles of freeze-thaw, storage at −80°C for 30 days, autosampler at 4°C for 24 h are as shown in Table 4. The RSD and RE ranges of the 14 compounds were 0.25–14.63% and −14.56–12.74%, respectively. The abovementioned data demonstrated that 14 compounds were all stable under different storage conditions.

### 3.3. Pharmacokinetic Study

Pharmacokinetic parameters reflected the changing rules of drug treatment process and could be used as a reference for clinicians to formulate an individual drug regimen for patients. Pharmacokinetic parameters in normal rats and model rats were calculated by DAS 2.0 software. The concentration-time curves of 14 compounds in normal rats and model rats are shown in Figure 4, and the corresponding pharmacokinetic parameters are presented in Table 5.

Caffeoylquinic acid compounds were absorbed quickly and reached to *C*_max_ within 1 h. Previous studies have shown that caffeoylquinic acid compounds were easily absorbed and metabolized in the intestine. When PH was neutral or alkaline, neochlorogenic acid and chlorogenic acid were easy to be transformed into cryptochlorogenic acid [32], and under the action of gut bacteria, chlorogenic acid is easy to be transformed into neochlorogenic acid and cryptochlorogenic acid [33]. Therefore, this may be the reason for the double peaks of neochlorogenic acid and cryptochlorogenic acid during four hours after administration APR. In addition, gut bacteria were disturbed and the intestinal PH changed under pathological conditions, which affected the isomerization of monosubstituted caffeoylquinic acid. Therefore, compared with normal rats, AUC_0-*t*_ and *C*_max_ of chlorogenic acid and cryptochlorogenic acid were increased, and longer *t*_1/2_ and MRT were observed in model rats. Meanwhile, there was no significant change in the pharmacokinetic parameters of neochlorogenic acid in normal and model rats, which may be due to the low participation and conversion of neochlorogenic acid in the isomerization of monosubstituted caffeoylquinic acid, and gut bacteria may have little effect on its absorption and metabolism.

For disubstituted caffeoylquinic acid, the gut bacteria changed under pathological conditions, which hindered the absorption of disubstituted caffeoylquinic acid by receptors on blood vessels, resulting in the AUC_0-t_ of 3,4-diCQA, 3,5-diCQA, and 4,5-diCQA being decreased. We speculated that the change of gut bacteria could also transform 3,4-diCQA and 4,5-diCQA into 3,5-diCQA, increasing the AUC_0-∞_, *C*_max_ and prolonging *t*_1/2_ of 3,5-diCQA. In addition, disubstituted caffeoylquinic acid could be hydrolyzed to monosubstituted caffeoylquinic acid by esterase produced by intestinal microorganisms such as colon bacillus, *Bifidobacterium* and *Lactobacillus gasseri*, or interconversion by esterase isomerization. This is also one of the main reasons for the inconsistent changes of pharmacokinetic parameters of disubstituted caffeoylquinic acid in arthritis rats, and its transformation mechanism remains to be further studied [34, 35].

For coumarin compounds, the 14 components could be detected in both normal and model rats 5 min after administration APR. The AUC_0-*t*_, AUC_0-∞_, and *C*_max_ of all compounds except columbianetin in model rats were higher than those in normal rats when given the same dose of the APR, which may be due to the effect of histamine being oversecreted by mast cells on receptors on blood vessels in model rats to increase vascular permeability, making coumarins easier to cross cell membranes and enter the blood [36]. Compared with normal rats, the *CL* of psoralen, bergapten, osthol, and columbianadin in model rats was decreased (*P* < 0.01), while the MRT_0-t_ of psoralen, bergapten, and columbianetin acetate was shortened (*P* < 0.01), which reflected the increased bioavailability of these compounds. The reasons may be (1) under pathological conditions, the activities of metabolic enzymes and transporters related to drug metabolism and transport in the body were changed, which significantly affected the *CL* of drug metabolized by the liver. (2) The active ingredients could prevent the diffusion of inflammation by affecting the binding of active ingredients to plasma proteins, inflammatory factors, and related receptors in the lesion of model rats, thus affecting the pharmacokinetics process of drugs in *vivo*. (3) The active ingredients were distributed to other tissues. (4) The active ingredients were transformed into other components under the action of gut bacteria and drug metabolism enzymes. In addition, for bergapten, the first peak appeared at 5 min after administration of APR and the second peak appeared at 4 hours, we speculated that the possible reason was as follows: xanthotoxin, an isomer of bergapten, which could transform to bergapten in a certain way in *vivo* so as to make the bergapten peak appeared again after dosing 4 h. For columbianetin acetate, the double peak phenomenon occurred in 4 h after administration of APR, which may be caused by the conversion of columbianetin into columbianetin acetate in *vivo* through liver metabolic enzymes or gut bacteria, or the hepatointestinal circulation. Furthermore, compared with normal rats, the AUC_0-*t*_, AUC_0-∞_, *C*_max_ of columbianetin decreased while *CL* increased and MRT shortened in model rats, which was consistent with our speculation.

In conclusion, compared with normal rats, the pharmacokinetic parameters of 14 compounds in normal and model rats were significantly different. This indicated that the pharmacokinetic behavior of drugs will vary with the pathological state of the body. This study found that the pharmacokinetic behavior of 14 components in APR was correlated with the pathological state of arthritis. This study provided important scientific information for better understanding the mechanism and clinical application of APR. At the same time, the abovementioned results also provide a scientific basis and data support for 14 compounds as a pharmacodynamic substance basis of APR against arthritis.

## 4. Conclusion

In this study, a UPLC-MS/MS method was established for simultaneous determination of 14 components in plasma and used to investigate the influence of arthritis induced by the complete Freund adjuvant on the pharmacokinetics of the14 components after oral administration of APR. The results showed that the established method had good accuracy, precision, recovery, and stability and was suitable for studying the pharmacokinetics of 14 components in rat plasma. In addition, there were significant differences in the pharmacokinetics of 14 compounds between normal and model rats. This suggested that it was necessary to formulate individualized and reasonable drug administration schemes according to different pathological states, which could not only effectively improve the safety and effectiveness of drugs but also reduce the probability of adverse reactions.

## Figures and Tables

**Figure 1:** The chemical structures of 14 compounds and ISs.

**Figure 2:** MDA and TNF-*α* levels in normal and model rats. (^*∗∗*^*P* < 0.01).

**Figure 3:** Chromatogram of blank plasma samples, blank plasma + LLOQ samples, and plasma samples of rats obtained from 5 min after administration ((A) neochlorogenic acid, (B) chlorogenic acid, (C) cryptochlorogenic acid, (D) 3,4-diCQA, (E) 3,5-diCQA, (F) 4,5-diCQA, (G) columbianetin, (H) psoralen, (I) xanthotoxin, (J) bergapten, (K) columbianetin acetate, (L) isoimperatorin, (M) osthol, (N) columbianadin, (O) chloramphenicol, and (P) daidzein).

**Figure 4:** Mean plasma concentration-time curves for (a) neochlorogenic acid, (b) chlorogenic acid, (c) cryptochlorogenic acid, (d) 3,4-diCQA, (e) 3,5-diCQA, (f) 4,5-diCQA, (g) columbianetin, (h) psoralen, (i) xanthotoxin, (j) bergapten, (k) columbianetin acetate, (l) isoimperatorin, (m) osthol, and (n) columbianadin in normal (black) and model (red) rats after oral administration of APR. (*n* = 6 of each group).

**Table 1:** The linear regression curve, correlation coefficient, and linear range of 14 compounds in rat plasma.

Analytes	Regression equation	R	Linear range (ng/mL)	LLOQ (ng/mL)
Neochlorogenic acid	*y* = 1.980*x* + 0.013	0.996	0.6–504	0.6
Chlorogenic acid	*y* = 1.842*x* + 0.054	0.992	10–3180	10
Cryptochlorogenic acid	*y* = 1.747*x* − 0.002	0.993	2.5–234	2.5
3,4-diCQA	*y* = 1.578*x* + 0.012	0.996	10.7–112	10.7
3,5-diCQA	*y* = 1.010*x* + 0.008	0.997	2.5–625	2.5
4,5-diCQA	*y* = 1.487*x* + 0.008	0.995	10.0–204	10.0
Columbianetin	*y* = 29.151*x* + 0.021	0.998	3.9–4520	3.9
Psoralen	*y* = 15.281*x* + 0.005	0.998	3.7–505	3.7
Xanthotoxin	*y* = 67.454*x* + 0.047	0.998	2.2–1120	2.2
Bergapten	*y* = 71.002*x* + 0.020	0.997	4.8–680	4.8
Columbianetin acetate	*y* = 2.499*x* − 0.008	0.998	7.4–4320	7.4
Isoimperatorin	*y* = 6.338*x* − 0.017	0.997	8.4–890	8.4
Osthol	*y* = 77.336*x* + 0.271	0.991	1.0–5500	1.0
Columbianadin	*y* = 0.536*x* + 0.014	0.996	6.4–2440	6.4

**Table 2:** Precision and accuracy of 14 compounds in rat plasma (*n* = 6).

Analytes	Concentration (ng/mL)	*Precision (RSD, %)*		*Accuracy (RE, %)*	
		Intraday	Interday	Intraday	Interday
Neochlorogenic acid	0.6	3.76	1.10	4.51	3.64
	10	4.00	9.21	4.21	10.86
	252	2.62	0.89	9.18	10.30
	504	8.31	13.52	2.38	10.70

Chlorogenic acid	10	6.72	4.99	0.75	0.05
	10.6	2.37	3.61	−6.49	−5.29
	1060	2.42	2.16	−2.73	−2.28
	3180	9.06	13.81	−14.76	−12.53

Cryptochlorogenic acid	2.5	4.33	0.99	3.58	2.49
	11.7	2.90	7.63	0.08	13.67
	117	2.97	2.92	5.04	3.55
	234	4.77	1.45	1.01	2.67

3,4-diCQA	10.7	9.33	1.40	4.55	6.19
	11.2	8.82	12.70	8.33	−0.36
	56	5.32	3.40	1.23	0.01
	112	0.82	0.17	5.30	4.83

3,5-diCQA	2.5	9.40	1.71	−1.56	−0.09
	12.5	6.15	5.84	5.17	9.80
	312.5	2.51	4.39	−3.79	−6.89
	625	1.06	2.62	0.61	2.14

4,5-diCQA	10.0	13.00	1.92	1.24	2.03
	20.4	3.17	1.42	−0.96	−0.26
	102	5.00	0.96	1.01	0.42
	204	1.20	2.44	1.36	0.03

Columbianetin	3.9	3.87	0.74	7.29	7.98
	39	8.72	4.37	9.64	6.70
	2260	1.24	3.77	3.63	5.96
	4520	0.72	0.94	−0.83	−0.34

Psoralen	3.7	2.18	2.43	0.27	2.72
	5.05	2.18	7.61	−9.26	13.01
	252.5	5.09	1.36	8.52	6.86
	505	2.73	2.61	7.39	9.30

Xanthotoxin	2.2	5.09	1.06	11.21	10.00
	11.2	6.02	5.90	0.14	3.41
	560	1.55	2.10	−1.18	−0.17
	1120	3.91	3.86	1.65	3.68

Bergapten	4.8	2.78	0.57	−0.95	−0.49
	13	8.09	4.08	9.96	5.18
	340	2.62	9.98	−8.05	−14.83
	680	6.81	3.61	12.28	9.14

Columbianetin acetate	7.4	8.11	1.56	−1.1	0.40
	54	7.45	1.88	4.31	3.04
	2160	1.86	4.52	5.87	5.73
	4320	3.47	1.98	4.25	6.62

Isoimperatorin	8.4	3.16	0.48	−3.08	−2.59
	8.9	0.39	1.74	1.87	2.19
	445	6.26	4.47	−13.39	−11.21
	890	5.63	4.77	2.76	4.52

Osthol	1.0	4.27	0.74	−3.96	−3.33
	5.5	7.70	4.21	−1.64	0.94
	2200	8.17	1.09	2.50	1.41
	5500	3.67	1.41	5.72	7.17

Columbianadin	6.4	14.22	2.09	11.09	13.84
	12.2	4.19	6.69	−10.37	1.22
	1220	9.14	1.66	3.43	1.91
	2440	8.07	2.82	4.83	7.40

**Table 3:** Recovery and matrix effect of 14 compounds and ISs in rat plasma (*n* = 6).

Analytes	Concentration (ng/mL)	*Recovery (%)*	*Matrix effect (%)*
		Mean ± SD	Mean ± SD
Neochlorogenic acid	10	98.37 ± 0.84	96.03 ± 0.24
	252	98.53 ± 1.18	97.36 ± 0.83
	504	99.35 ± 0.56	96.67 ± 0.71

Chlorogenic acid	10.6	93.79 ± 4.36	96.75 ± 0.60
	1060	98.67 ± 1.81	99.66 ± 0.40
	3180	99.55 ± 2.08	100.19 ± 2.90

Cryptochlorogenic acid	11.7	96.62 ± 0.81	95.87 ± 1.31
	117	93.56 ± 2.76	92.87 ± 2.47
	234	97.11 ± 1.50	93.64 ± 5.02

3,4-diCQA	11.2	96.45 ± 2.84	94.87 ± 4.77
	56	100.55 ± 1.03	94.29 ± 3.61
	112	94.39 ± 2.53	98.10 ± 0.79

3,5-diCQA	12.5	100.24 ± 1.44	99.19 ± 0.76
	312.5	99.44 ± 0.34	98.73 ± 1.47
	625	96.17 ± 2.42	93.75 ± 1.53

4,5-diCQA	20.4	95.94 ± 5.51	94.74 ± 5.71
	102	90.38 ± 7.27	88.11 ± 5.31
	204	98.24 ± 2.58	96.54 ± 1.30

Columbianetin	39	100.61 ± 1.72	91.94 ± 9.71
	2260	94.77 ± 4.24	94.89 ± 4.41
	4520	99.57 ± 0.56	99.45 ± 0.71

Psoralen	5.05	93.25 ± 4.57	96.85 ± 0.22
	252.5	96.67 ± 6.07	98.33 ± 1.58
	505	99.16 ± 0.67	98.98 ± 0.53

Xanthotoxin	11.2	97.27 ± 1.08	98.69 ± 1.27
	560	97.90 ± 1.24	98.17 ± 0.99
	1120	95.60 ± 0.47	99.72 ± 0.11

Bergapten	13	94.7 ± 9.98	95.13 ± 9.57
	340	103.73 ± 2.78	92.19 ± 8.08
	680	100.62 ± 10.70	96.77 ± 8.80

Columbianetin acetate	54	95.58 ± 0.88	93.72 ± 6.68
	2160	98.04 ± 1.90	100.09 ± 7.76
	4320	100.06 ± 3.49	97.66 ± 3.34

Isoimperatorin	8.9	99.29 ± 2.11	99.81 ± 1.91
	445	95.01 ± 3.06	95.95 ± 2.76
	890	95.66 ± 5.42	90.78 ± 9.05

Osthol	5.5	94.26 ± 3.63	96.24 ± 0.79
	2200	99.93 ± 1.34	98.92 ± 2.45
	5500	100.16 ± 1.59	98.70 ± 0.70

Columbianadin	12.2	91.42 ± 3.26	94.17 ± 5.35
	1220	99.66 ± 1.20	99.85 ± 1.67
	2440	96.46 ± 9.48	102.29 ± 8.50

Chloramphenicol	100	96.68 ± 2.07	97.72 ± 3.17
Daidzein	100	99.74 ± 6.36	99.75 ± 1.89

**Table 4:** The stability test of 14 compounds in rat plasma (*n* = 6).

Analytes	Concentration (ng/mL)	*Short term stability*		*Long term stability*		*Freeze-thaw cycles stability*		*Posttreatment stability*	
		RSD (%)	RE (%)	RSD (%)	RE (%)	RSD (%)	RE (%)	RSD (%)	RE (%)
Neochlorogenic acid	10	2.83	3.18	3.80	3.30	4.30	2.40	7.71	0.96
	252	4.02	11.46	4.33	11.71	2.86	10.25	2.10	9.31
	504	12.07	3.48	13.42	1.97	11.60	2.89	10.32	3.01

Chlorogenic acid	10.6	13.41	−10.70	11.16	−10.10	9.30	−9.38	7.04	−8.90
	1060	0.57	−4.07	2.31	−3.00	0.96	−7.72	2.42	−2.64
	3180	2.98	−12.94	5.95	−14.43	11.29	−14.56	8.15	−12.93

Cryptochlorogenic acid	11.7	4.62	0.09	7.81	0.11	4.91	0.10	2.47	0.05
	117	5.89	2.98	5.10	2.57	4.78	2.12	3.40	2.21
	234	7.76	3.55	8.13	1.12	6.02	0.54	5.95	0.37

3,4-diCQA	11.2	9.42	7.83	8.78	8.03	11.50	4.70	10.99	3.59
	56	3.26	1.26	5.41	0.47	2.76	0.11	2.41	2.38
	112	11.76	10.17	11.25	9.46	6.54	12.74	8.70	10.42

3,5-diCQA	12.5	2.91	10.66	7.37	5.53	2.47	11.59	6.67	2.20
	312.5	7.18	−2.48	6.17	−3.61	5.56	−3.62	4.84	−3.41
	625	2.51	1.54	2.33	1.49	2.15	1.58	1.80	1.31

4,5-diCQA	20.4	5.56	−0.05	5.22	−1.39	4.65	−1.10	4.61	−1.17
	102	3.52	1.81	4.46	1.98	4.57	1.74	2.78	0.33
	204	2.03	0.82	1.41	0.18	1.67	0.80	1.81	0.03

Columbianetin	39	5.28	0.47	4.79	8.79	1.88	−5.49	2.58	7.89
	2260	3.07	4.19	2.27	3.56	1.39	3.82	1.55	3.59
	4520	1.27	−0.87	1.18	−0.94	0.98	−0.84	0.86	−0.88

Psoralen	5.05	5.69	−5.85	3.17	−8.84	10.07	−8.37	1.57	−13.10
	252.5	3.86	7.43	5.16	9.22	0.45	11.50	1.70	5.27
	505	5.47	7.62	4.56	5.91	0.93	10.13	2.53	8.21

Xanthotoxin	11.2	9.77	0.18	9.36	−0.74	7.04	0.06	7.03	−0.52
	560	2.68	−0.81	2.57	−0.76	2.16	−0.74	1.97	−1.16
	1120	2.36	7.30	2.76	7.34	4.24	6.75	4.79	1.28

Bergapten	13	6.95	0.63	7.66	1.53	7.64	2.72	8.44	1.62
	340	9.35	−13.21	6.41	−12.79	6.19	−7.04	3.46	−10.30
	680	7.50	5.28	4.17	1.84	7.17	4.19	6.40	7.29

Columbianetin acetate	54	8.01	0.55	7.18	2.56	7.42	1.77	2.03	1.96
	2160	7.73	7.96	5.53	3.76	6.37	9.80	0.25	6.87
	4320	3.35	2.64	1.90	3.38	4.58	4.44	4.29	4.02

Isoimperatorin	8.9	2.74	1.35	4.79	0.03	3.83	1.05	1.78	0.78
	445	2.83	−12.34	3.49	−12.65	4.33	−13.11	5.87	−13.01
	890	2.60	0.18	6.96	0.87	4.10	0.53	3.37	1.16

Osthol	5.5	0.73	3.44	6.79	-0.08	4.39	−3.84	3.64	−3.39
	2200	4.19	0.28	8.56	0.09	2.82	0.81	4.34	1.27
	5500	2.27	0.82	4.58	0.53	5.89	1.74	2.70	5.18

Columbianadin	12.2	14.15	−2.01	12.98	−1.51	14.63	−8.53	13.80	−6.29
	1220	7.48	2.07	7.02	1.08	8.37	−0.74	6.79	0.72
	2440	9.13	−5.05	6.13	−2.67	8.24	−0.12	9.69	−2.46

**Table 5:** The main pharmacokinetic parameters of 15 compounds in normal and arthritic model rat groups after oral administration of APR (mean ± SD, *n* = 6).

Analytes	Group	AUC_0-*t*_ (ng/L^*∗*^h)	AUC_0-∞_ (ng/L^*∗*^h)	*C*_max_ (ng/mL)	*t*_max_ (h)	*t*_1/2_ (h)	MRT_0-*t*_ (h)	*CL* (L/h/kg)
Neochlorogenic acid	Normal	1140.97 ± 76.91	1841.89 ± 375.29	419.76 ± 58.64	0.20 ± 0.04	39.94 ± 16.54	15.59 ± 0.68	16.79 ± 3.08
	Model	1191.17 ± 45.24	1730.83 ± 234.76	531.12 ± 24.05	0.23 ± 0.03	31.80 ± 10.17	15.60 ± 0.26	17.56 ± 2.06

Chlorogenic acid	Normal	3750.55 ± 258.95	5361.78 ± 591.80	1669.61 ± 25.80	0.54 ± 0.36	27.89 ± 14.85	5.95 ± 0.28	5.64 ± 0.56
	Model	4518.22 ± 123.41^*∗∗*^	5658.96 ± 1752.92	2759.25 ± 264.26^*∗∗*^	0.45 ± 0.10	51.97 ± 13.17^*∗*^	8.68 ± 0.52^*∗∗*^	5.67 ± 1.47

Cryptochlorogenic acid	Normal	1293.94 ± 31.4	2023.36 ± 571.79	142.61 ± 4.63	0.42 ± 0.12	34.55 ± 17.65	18.26 ± 0.46	15.70 ± 3.89
	Model	1695.03 ± 117.262^*∗∗*^	3849.34 ± 472.22^*∗∗*^	188.64 ± 8.70^*∗∗*^	0.45 ± 0.10^*∗∗*^	48.36 ± 10.53	19.51 ± 0.55^*∗∗*^	7.89 ± 1.02^*∗∗*^

3,4-diCQA	Normal	664.51 ± 54.19	1472.35 ± 280.50	85.71 ± 8.14	0.29 ± 0.10	57.97 ± 11.96	21.16 ± 0.73	21.06 ± 4.38
	Model	504.41 ± 19.59^*∗∗*^	1744.69 ± 748.99	79.74 ± 7.11	0.29 ± 0.10	84.47 ± 24.30^*∗*^	19.81 ± 0.40^*∗∗*^	19.66 ± 7.70

3,5-diCQA	Normal	1129.67 ± 137.54	1762.50 ± 613.93	292.78 ± 47.74	0.18 ± 0.03	33.90 ± 14.30	21.07 ± 0.68	18.37 ± 4.81
	Model	961.07 ± 40.95^*∗*^	3223.71 ± 110.12^*∗*^	405.33 ± 49.16^*∗∗*^	0.18 ± 0.03	59.48 ± 17.24^*∗*^	18.79 ± 0.49^*∗∗*^	10.62 ± 4.85^*∗*^

4,5-diCQA	Normal	1011.06 ± 30.37	2283.82 ± 375.11	125.50 ± 11.99	0.24 ± 0.03	52.82 ± 19.30	21.70 ± 0.72	11.34 ± 6.62
	Model	760.23 ± 40.08^*∗∗*^	1287.79 ± 198.07^*∗*^	154.10 ± 8.92^*∗∗*^	0.23 ± 0.03	40.72 ± 5.72^*∗∗*^	21.72 ± 0.78	11.76 ± 9.60

Columbianetin	Normal	30285.36 ± 1540.07	30618.34 ± 1524.53	3116.03 ± 241.95	9.67 ± 0.82	6.04 ± 0.12	13.30 ± 0.36	0.98 ± 0.05
	Model	25928.65 ± 675.38^*∗∗*^	26123.62 ± 692.36^*∗∗*^	2220.70 ± 167.90^*∗∗*^	9.00 ± 1.09	6.07 ± 1.28	12.10 ± 0.20^*∗∗*^	1.14 ± 0.03^*∗∗*^

Psoralen	Normal	3231.02 ± 159.33	3431.94 ± 240.22	209.65 ± 27.61	8.00 ± 1.26	9.80 ± 3.28	14.34 ± 0.31	8.77 ± 0.59
	Model	3745.47 ± 90.89^*∗∗*^	3770.10 ± 922.58^*∗∗*^	326.62 ± 42.49^*∗∗*^	7.66 ± 0.81	5.98 ± 0.44^*∗*^	12.93 ± 0.22^*∗∗*^	7.96 ± 019^*∗∗*^

Xanthotoxin	Normal	4443.85 ± 187.58	4619.69 ± 224.28	553.93 ± 76.03	4.33 ± 0.82	12.12 ± 1.73	10.72 ± 0.53	6.50 ± 0.31
	Model	4637.98 ± 148.45	4887.81 ± 179.48^*∗*^	528.00 ± 34.98	3.33 ± 1.03	14.25 ± 3.76	10.30 ± 0.51	6.14 ± 0.22

Bergapten	Normal	2263.69 ± 175.96	2331.37 ± 183.83	383.01 ± 95.75	3.67 ± 0.82	9.41 ± 2.12	9.40 ± 0.34	12.93 ± 1.05
	Model	3119.18 ± 100.34^*∗∗*^	3185.02 ± 140.89^*∗∗*^	518.44 ± 42.86^*∗*^	4.67 ± 1.03	7.16 ± 0.41	7.11 ± 0.09^*∗∗*^	9.43 ± 0.42^*∗∗*^

Columbianetin acetate	Normal	9066.10 ± 950.05	10092.04 ± 1428.28	2020.33 ± 162.24	0.18 ± 0.03	17.30 ± 3.61	18.56 ± 0.64	2.61 ± 1.06
	Model	9190.51 ± 376.09	10597.06 ± 389.11	2243.01 ± 304.11	0.15 ± 0.03	15.92 ± 2.06	15.83 ± 0.91^*∗∗*^	2.83 ± 0.10

Isoimperatorin	Normal	1188.60 ± 68.55	1555.48 ± 149.22	224.37 ± 26.80	0.58 ± 0.20	26.91 ± 8.34	15.10 ± 0.57	19.42 ± 1.73
	Model	1277.40 ± 36.97^*∗*^	1653.04 ± 86.14	232.11 ± 20.96	0.58 ± 0.20	26.76 ± 5.46	15.71 ± 0.65	18.18 ± 0.88

Osthol	Normal	11448.25 ± 552.50	11648.88 ± 567.74	3642.21 ± 286.50	1.16 ± 0.40	13.42 ± 0.51	6.53 ± 0.29	2.58 ± 0.11
	Model	22518.30 ± 2167.96^*∗∗*^	22544.07 ± 2169.73^*∗∗*^	4561.27 ± 271.63^*∗∗*^	0.91 ± 0.20	6.42 ± 0.69^*∗∗*^	6.94 ± 0.42	1.33 ± 0.11^*∗∗*^

Columbianadin	Normal	2661.55 ± 122.95	2968.16 ± 200.66	1683.74 ± 221.50	0.23 ± 0.03	16.43 ± 3.96	12.30 ± 0.57	10.14 ± 0.70
	Model	3487.92 ± 132.71^*∗∗*^	3849.07 ± 265.00^*∗∗*^	1497.02 ± 48.21	0.23 ± 0.03	16.51 ± 4.83	11.51 ± 0.87	7.82 ± 0.51^*∗∗*^

^*∗*^ *P* < 0.01 and ^*∗∗*^*P* < 0.01 compared with the normal group.

## Data Availability

The data used to support the findings of this study are included within the article.
